The article "The impact of FDI on the agriculture sector: A case study from Bangladesh" was retracted in 2025. Reasons: suspected computer-generated content; unreliable results or conclusions.

# The impact of FDI on the agriculture sector: A case study from Bangladesh

**DOI:** 10.1016/j.heliyon.2023.e22983

**Published:** 2023-11-28

**Authors:** Zakia Sultana, Md Nazmus Sadekin

**Affiliations:** Department of Economics, Mawlana Bhashani Science and Technology University, Santosh, Tangail-1902, Bangladesh

**Keywords:** Agricultural sector, ARDL, Bangladesh, Devaluation, F-bound test, Foreign direct investment

## Abstract

This paper aims to inspect the relationship between Foreign Direct Investment (FDI) and the agricultural sector of Bangladesh. This study is based on time series data from 1972 to 2021. The Auto Regressive Distributed Lag (ARDL) model and F-Bound test are used to examine the relationship between the variables under study. The empirical finding suggests that FDI has a considerable negative influence on the agricultural sector in Bangladesh in the long term. Moreover, this is also found by the study that FDI has no effect in the short run on the country's agricultural sector. This study recommends that governments should adopt agriculture-friendly policies, and should adopt some training facilities for the farmer to increase their farming skills so that FDI can develop the agricultural sector.

## 1 Introduction

At present Foreign Direct Investment (FDI) is an important issue in many aspects for a country. In developing countries like Bangladesh, FDI plays a vital role [1]. It is a vital source of income and a possible lifeline for many developing countries, specifically where poverty, savings, and unemployment rates are high [2]. According to government estimation, about 14 % of the population in Bangladesh is still living below the poverty line in the 2021–2022 fiscal year [3] [BBS]. Foreign Direct Investment [FDI] helps to build up different sectors [4], Agricultural sector is one of them. Developing economies must expand their investment in agriculture [1]. Even though Bangladesh is endowed with agriculturally productive land, food insecurity, and scarcity have been issues across the continent. Bangladesh needs to expand and expedite investment. According to [BBS] Bangladesh is an agriculture-based country. With 156.8 million people (BBS, 2014), it has the highest population density in the world, with 1063 people per square kilometer, 66 % of people live in rural areas. Agriculture is the main workforce for 45 % of the population. More than 14.74 % of the GDP is contributed by agriculture. Crops, livestock, fisheries, and forests are just a few of the diverse subsectors that make up this sector, and that is 55 %, 14 %, 22 %, and 9 % of its agricultural economy, correspondingly [5]. Bangladesh's economy has always been dominated by agriculture. The majority of the people live in rural areas, where agriculture is their principal source of income. "Agricultural development is the source of the country's entire economic progress," stated Muhammad Abdur Razzaque, Bangladesh's agriculture minister. The agriculture sector contributes 12.09 % to the GDP [3]. According to [Bangladesh Investment Development Authority] the agricultural sector produces around 70 million metric tons of output, primarily rice, potatoes, and sugar crops, and FDI oversees and promotes private investment. Around 700 kinds of goods to over 140 countries are exported by Bangladesh, the majority of which are cereal grains, processed meat, vegetables, tobacco, cut flowers, frozen fish, fruits, tea, spices, dry food, and other processed agricultural products such as cow, chicken, and fish feed. 35 % of exports are made up of four agricultural items [6]. Agriculture accounted for 12.09 % percent of Bangladesh's gross domestic GDP (BBS, 2020–2021). Industry made up around 34.61 % percent of the total, while the services sector made up about 53.30 % [3]. The agriculture sector's contribution to the economy is small compared to other sectors [4]. A crucial tactic for fostering economic growth and development in a developing nation like Bangladesh is foreign direct investment. FDI can stimulate economic expansion. It enhances the likelihood that a nation will develop its integration into international financial flows, grow its exports and employment base, and produce technical spillovers of efficiency and capacity-building to domestic businesses [7]. FDI offers an investment structure that boosts economic growth. For many developing nations, notably Bangladesh, where there is a high rate of poverty, little culture of saving, and weak or nonexistent financial markets, foreign direct investment (FDI) is a significant source of funding and a possible lifeline [8]. Additionally, several scholars have emphasized the significance of FDI for the expansion of the economies of the host countries, whether by augmenting local capital to foster expansion or by having an effect through the transfer of technology and expertise. These advantages of FDI have encouraged many nations, particularly developing nations, to implement laws and other incentives to draw FDI from abroad [9]. Numerous empirical research on the relationship between FDI and growth have been conducted to better understand whether these inflows benefit the host economies [10]. While some have looked at how FDI may supply domestic capital formation, others have examined how FDI can have spillover effects. Many have focused their research on the way that FDI affects the host country's economic growth. If raising the FDI inflow in the agriculture sector it will create more economic development. A country's FDI and Agriculture have a direct and tangled relationship. Bangladesh's economy is still dependent on agriculture. Investment in various sectors of a country is essential to improve a developing country's financial development. In this age of globalization, the FDI provides an amazing opportunity for developing countries to achieve faster monetary development [11]. FDI is one of the most important components for increasing job prospects in the agriculture sector through commercialization and modernization, as the industry employs 52 % of the workforce. FDI has become a major engine of economic growth and development in industrialized countries for the past two decades. Even in underdeveloped and less developed countries, the FDI can accelerate the growth of the economy. Moreover, Foreign Direct Investment (FDI) can help to develop human resources, domestic production, and infrastructure [2]. Bangladesh may have some successful mechanisms in place to preserve foreign direct investment and guarantee a pleasant environment in which to invest. That means to boost Bangladesh's economic growth, new tactics for attracting inward FDI should be implemented.

According to Fig. 1, we can see the sector-wise net FDI inflow of Bangladesh in fiscal year 2019–20. The contribution of FDI in the agricultural sector is about 0.5 %. Compared with other sectors this contribution is very poor [12].

**Fig. 1:** Sector-wise net inflow FY 2019–20.

Source [12]:

However, agriculture continues to be Bangladesh's main source of income, although the country's modern economy is mostly dependent on industrialization. In Bangladesh, agriculture has frequently served as a driving force behind long-term success and development. The agriculture industry is still the country's most important source of economic growth. Bangladesh's economy can grow because of the effectiveness of foreign direct investment, and it can help the government to meet its socioeconomic goals, including poverty reduction targets [8]. In a developing country like Bangladesh, FDI can be an important component for increasing productive resources and creating job opportunities and also has a positive as well as significant impact on GDP [13].

Rural areas are where the bulk of the world's poor reside. For 84 % of rural residents, agriculture is their primary means of subsistence [14]. Farming systems frequently involve a variety of interconnected gathering, production, and post-harvest processes, so in addition to farming, rural households may also engage in a variety of activities related to livestock, agro-forestry, fishing, and aquaculture as well as other important agricultural sub-sectors. The agricultural sector in Bangladesh is divided into various sub-sectors such as production, animal, forestry, and fisheries. 12.09 % of GDP is shared by the Agricultural sector, including fishing at 11 %, crops, and horticulture at 55 %, animal and farming at 18 %, and forest and related services at 16 % [3]. Bangladesh is facing many problems, one of them is poverty. “The lower level of investment leads to a lower level of productivity when the productivity per worker is low, the real income will be low and so there poverty and the vicious circle is complete” [15]. The importance of agricultural development in eliminating vicious circulation is immense [16]. Foreign Direct Investment is one of the ways, in which agricultural development can be enhanced. At present FDI inflow in Bangladesh is 2.37 (FY20), and the FDI inflow in the agriculture sector is much less than the other countries. If we can increase FDI inflow in the agriculture sector then poverty reduction may be possible [10]. The rate of contribution to agricultural growth is 52 %. Hunger affects about 800 million people worldwide, the large majority of whom reside in underdeveloped countries (United Nations, 2015) [17]. Bangladesh received $16.9 billion in foreign direct investment in 2019 (FDI). The United States is the leading investor, with $ 3.5 billion in net assets. Bangladesh attracted $1.6 billion in foreign direct investment in 2019. Foreign direct investment (FDI) inflows were barely 0.53% of GDP, one of Asia's lowest rates. Despite the government's efforts to provide a flexible and accommodating climate, the agriculture industry remains an unattractive and unprofitable sector for FDI in Bangladesh. In comparison to other sectors, agriculture receives less attention, than industries, and services.

The study will determine the answers to the following questions**:** What is the relationship between FDI and the Agriculture sector in Bangladesh? What is the effect of Foreign Direct Investment on the Agricultural sector? We anticipate that our research will shed additional light on the nature of Bangladesh's agricultural sectors, in connection with foreign direct investments. In addition, the primary goal of this research is to identify the factors that influence foreign direct investment (FDI) in the agricultural sector in developing nations like Bangladesh. The main objective of this study is to inspect the relationship between FDI and the agricultural sector in Bangladesh.

## 2 Conceptual framework & literature review

### 2.1 Operational definition of FDI

According to the OECD Benchmark Definition of Foreign Direct Investment, “Foreign direct investment reflects the objective of obtaining a lasting interest by a resident entity in one economy (‘‘direct investor’’) in an entity resident in an economy other than that of the investor (‘‘direct investment enterprise’’). The lasting interest implies the existence of a long-term relationship between the direct investor and the enterprise and a significant degree of influence on the management of the enterprise.” Direct investment covers not only the initial transaction but also all subsequent capital transactions between them and among associated enterprises including both incorporated and unincorporated [18]. According to Ref. [19], FDI can be categorized into the following five types: a) Mergers and acquisitions, b) Joint Venture, c) Horizontal FDI, and d) Vertical FDI.

According to Ref. [20] Foreign direct investment (FDI) is a powerful tool for growing the Bangladeshi economy and can help the nation achieve its socioeconomic goals, including poverty reduction. Bangladesh, a nation with little access to capital, FDI has the potential to become a substantial tool for increasing physical capital and creating jobs, and possibilities, increasing productive capacity, and improving local workers' skills through transferring and managing expertise, and assisting in integration the local economy with the worldwide economy.

### 2.2 Agriculture sector

Bangladesh, with a geographical size of 1,47,570 square kilometers, is one of the world's most agro-based underdeveloped countries [21]. Agriculture has long been a necessary part of Bangladesh's economy. Agricultural development plays a vital role in removing poverty reduction and country development. Without the agricultural development of a country, development cannot be imagined. According to Ref. [15] Agricultural sector is divided into some sub-sectors such as (Life stock, Farming, Forestry, and Fishing).

### 2.3 Empirical literature review

According to Ref. [22], to examine the relationship between FDI and the Agricultural sector in Nigeria using quarterly time series data for the period 1981–2017 based on the autoregressive distributed lag (ARDL) model, they suggested that the output of the agricultural sector is positively and significantly influenced by the foreign direct investment. The ARDL result specifically demonstrates that the impact of foreign direct investment is greater in the near term than in the long term. Additionally, across the study period, economic deregulation had a considerable impact on agricultural output [9]. Discuss the impact of FDI on the agricultural sector in country Ghana. Using data from 1980 to 2013 and the Johansen cointegration test, they examined the effects of FDI on the performance of the agricultural sector in Ghana. We discovered that FDI has a long-term, negative influence on agricultural sector production, but a short-term, positive association.

[23]In this study, it is examined the relationship between Nigeria's economic growth and foreign direct investment (FDI). Bound testing and the Autoregressive Distributed Lags (ARDL) model are used to estimate data for the years 1981 through 2013. Results demonstrated that FDI and economic growth have a long-term (cointegrating) link. Their statistically meaningful negative error correction model had an error correction of roughly 43 %. FDI has a tiny, negligible impact on growth in the short term and a small, negligible impact on growth in the long term [24].they analyze the variables (VAR) model which was utilized using a three-step process to assess the impacts of FDI, trade, and its effects on agricultural sector development in Nigeria between the years of 1980–2009. The results of the Granger causality test indicate that there is no causal relationship, a bidirectional relationship, and a unidirectional relationship between the variables used.

[11] They investigate how FDI affects the Indian economy's agricultural sector and look at its effects. They show an inverse relationship between FDI growth and the agriculture sector [25]. Their article simulates the economy by enhancing company confidence using an 86-sector computable general equilibrium model of Bangladesh. It discovered that rural households have lower consumption, as a result of their concentration on the agricultural industry, which is negatively impacted [26]. The aim is to find out the relationship between FDI and agricultural growth in Nigeria from 1981 to 2014 using annual time series data. The association between agricultural growth and FDI in agriculture was positive but nonsignificant, indicating that the factor directly neither affects agricultural growth nor obscures its effect by other macroeconomic factors [27]. Examine the impact of foreign direct investment (FDI) on land in developing countries' agriculture, Found the descriptive analysis that there is a difference in the influence on the host countries' food security.

[28] By analyzing the short- and long-term impacts of different sectors' productivity on economic growth in the South African district using a panel autoregressive distributed lag model (ARDL). Using yearly data from 1996 to 2015, According to the findings, productivity in the manufacturing, commerce, construction, transportation, and financial sectors has a beneficial long-term impact on economic growth. The productivity of the mining and tourist industries, however, has a long-term negative effect on economic growth. According to short-run statistics, every sector's productivity aside from commerce and transportation contributes favorably to local economic growth in the short term. According to Ref. [29], Both linear and non-linear panel autoregressive distributive lag (panel ARDL) models are used to support their estimate. The symmetric model was proven to have a favorable and large long-term influence on economic growth using an annual dataset from 1990 to 2018. However, the short-term projections indicate that the oil price has little to no effect on economic expansion. The overall outcomes of the asymmetric model also demonstrate that the link between the price of oil and economic development in the examined nations is non-linear.

## 3 Methodology

### 3.1 Methodology and research design

The purpose of the research design is to provide an acceptable framework for a study. An important phase in the research design process is deciding on a research approach, which determines how relevant data for a study, will be acquired. Based on secondary data collecting, various types of graphs and tables (using Microsoft Word, Microsoft Excel, and Strata software) are applied in this research. The secondary data is generally collected from journal papers, official documents, books, articles, thesis papers, daily newspapers, etc. For the study, our research paper data were collected from the World Development Indicator.

### 3.2 Framework

The materials for this study, have been collected from WDI data spanning the years 1972–2021, for analyzing our objectives. These are the grounds for selecting these times is the availability of data. The variables that have been used as the independent variables are Foreign Direct Investment, Employment in the Agriculture Sector, Inflation, Gross Fixed Capital Formation, Gross Domestic Product, and Trade, and the dependent variable is the agriculture sector (Forestry, Fisheries). Above the 6 variables, 4 have been chosen, as in previous literature [9] and GDP has been chosen because Previous literature suggested that GDP and FDI had a positive relationship. According to Ref. [20] a positive relationship exists between FDI and GDP and one variable Employment in the agriculture sector is suggested by the Authors. The sample of data used for econometric investigation will be based on 50 years of data collected every year for objectives.

### 3.3 Data collection method

Data was collected for our two objectives from WDI and their period is 1972–2021. The details of the data are given in Table 1.

**Table 1:** Functional relationship and source of data.

Name of Variables	Types of Variables	Abbreviation	Source of Data	Time
Agriculture (Forestry and Fisheries)	Dependent variable	AFF	WDI	1972–2021
Foreign Direct Investment	Independent variable	FDI	WDI	1972–2021
Employment in Agriculture	Independent variable	EIG	WDI	1972–2021
Gross Fixed Capital Formation	Independent variable	GFCF	WDI	1972–2021
Gross Domestic Product	Independent variable	GDP	WDI	1972–2021
Inflation (Consumer price annual)	Independent variable	CPI	WDI	1972–2021
Trade	Independent variable	Trade	WDI	1972–2021

### 3.4 Model specification

The study's focus is to find out the relationship between FDI and the Agriculture sector. ARDL is used for achieving the objective of the study, and similar types of models are used by Ref. [9] to discuss the impact of FDI on the agricultural sector in country Ghana. Especially [22] used the ARDL model to determine the impact of FDI on the Agriculture sector in Nigeria and [24,30]**.** Here use a similar (ARDL) model.

### 3.5 Econometric model estimation

In the agricultural sector in this model, the output is defined as a function of foreign direct investment (FDI), inflation (CPI), Employment in Agriculture (EIG), Trade Openness (TRADE), Gross Fixed Capital Formation Expressed as a % of GDP (GFCF) and Gross Domestic Product (GDP). Our investigation focuses on employing bounds testing of co-integration and autoregressive distributed lag (ARDL) models to examine the long-run relationship between the variables of interest. To determine if the lagged values of variables in an unlimited error correction regression are significant, Bounds tests, construct a Wald statistic [31]. The chosen method of analysis is justified by the fact that, in contrast to Engle and Granger's (1987) single equation method, it permits the testing of co-integrating connection hypotheses. Second, besides other techniques for examining long-term relationships, the Bounds method does not impose rigid limitations on the variables' integrating order. Lastly, it is a more effective method for evaluating co-integration. Our Bounds-test is in Equation (1).

(1) $$\Delta {AFF}_{t}=\beta_{0}+\beta_{1}\sum_{1=i}^{q}{\Delta AFF}_{t-i}+\beta_{2}\sum_{1=i}^{q}{\Delta FDI}_{t-i}+\beta_{3}\sum_{1=i}^{q}{\Delta EIG}_{t-i}+\beta_{3}\sum_{1=i}^{q}{\Delta GDP}_{t-i}+\beta_{4}\sum_{1=i}^{q}{\Delta CPI}_{t-i}+\beta_{5}\sum_{1=i}^{q}{\Delta TRADE}_{t-i}+\beta_{6}\sum_{1=i}^{q}{\Delta GFCF}_{t-i}+\alpha_{1}{AFF}_{t-i}+\alpha_{2}{FDI}_{t-i}+\alpha_{3}{EIG}_{t-i}+\alpha_{4}{GDP}_{t-i}+\alpha_{5}{CPI}_{t-i}+\alpha_{6}{TRADE}_{t-i}+\alpha_{7}{GFCF}_{t-i}+\varepsilon_{t}$$

Here $\beta_{0}$ is intercept and $\varepsilon_{t}$ is stochastic term respectively, while Δ is the difference operator for the lagged values of the variable's beta (β) shows short run and alpha (α) shows long run relationship.

The null hypothesis suggests that a long-term association is not present. To assess the importance of the lagged values of variables in an unconstrained error correction regression, the test calculates an F-statistic [30].

Additionally, the lower bound and upper bound asymptotic critical values are computed. The upper bound critical value is based on the assumption that all regressors are I, whereas the lower bound critical value is based on the assumption that all causative variables are I(0) (1). If the F-statistic is higher than the critical value at the upper bound, which suggests a long-run link exists, the null hypothesis that there is no association between the levels of the variables is rejected. On the other hand, if the F- statistic is smaller than the critical value at the lower bound, indicating that no long-run association exists, the null would not be rejected. However, if this statistic is within the two boundaries, the test is inconclusive, and before we can draw any findings, we must know more about the sequence of integration of each of the variables [30]. In the 2nd step, the long-run and short-run models are implied by Equation (2) and Equation (3).

(2) $$\Delta {AFF}_{t}=\alpha_{0}+\alpha_{1}{AFF}_{t-i}+\alpha_{2}{FDI}_{t-i}+\alpha_{3}{EIG}_{t-i}+\alpha_{4}{GDP}_{t-i}+\alpha_{5}{CPI}_{t-i}+\alpha_{6}{TRADE}_{t-i}+\alpha_{7}{GFCF}_{t-i}+\varepsilon_{t}$$

(3) $$\Delta {AFF}_{t}=\beta_{0}+\beta_{1i}\sum_{1=i}^{q}{\Delta AFF}_{t-i}+\beta_{2i}\sum_{1=i}^{q}{\Delta FDI}_{t-i}+\beta_{3i}\sum_{1=i}^{q}{\Delta EIG}_{t-i}+\beta_{4i}\sum_{1=i}^{q}{\Delta GDP}_{t-i}+\beta_{5i}\sum_{1=i}^{q}{\Delta CPI}_{t-i}+\beta_{6i}\sum_{1=i}^{q}{\Delta TRADE}_{t-i}+\beta_{7i}\sum_{1=i}^{q}{\Delta GFCF}_{t-i}+\varphi {ECM}_{t-i}+\varepsilon_{t}$$

Here φ is the error correction coefficient. The researcher employed the use of Stata econometric software for the data analysis.

## 4 Empirical results and discussions

### 4.1 Unit root test

We used the Augmented Dickey-Fuller (ADF) test to determine whether each data series is integrated and has a unit root before moving on to the ARDL bound test. A variable with a unit root is non-stationary in the level from but turns stationary after being differenced, hence testing the stationary of these time series.

Some of the variables mentioned in Table 2 are non-stationary at the same levels, which necessitates the next step of differentiating the non-stationary variables once before doing a stationary test on the differentiating variables. Following differencing, the data (See: Table 2) demonstrate that all of the variables are reliably stationary. To support the use of the Autoregressive Distributed Lag (ARDL) technique to co-integration because it (See: Table 2) gives mixed results.

**Table 2:** Unit root test result.

Variables	At the levels		After first difference		Decision
Test Statistics		Stationary Position	Test Statistics	Stationary Position	
LnAFF	−0.0283545	Not Stationary	−1.048584	Stationary	I (1)
FDI	−.1114829	Not Stationary	−1.156586	Stationary	I (1)
EIG	−0.839077	Not Stationary	−0.9918224	Stationary	I (1)
GDP	−0.9892071	Stationary	−1.274356	Stationary	I (0)
CPI	−0.2956979	Stationary	−1.248505	Stationary	I (0)
TRADE	−0.0829524	Not Stationary	−0.7136264	Stationary	I (1)
GFCF	−0.1261184	Not Stationary	−1.272271	Stationary	I (2)

### 4.2 Test for co-integration relationship

Once the variables’ stationary has been established, we investigate whether or not the variables' co-integration is present. When a co-integration relationship exists, it indicates that the long-run equilibrium and trend are shared by all seven of the variables used, as theorized. However, the results of the unit root tests allow us to estimate an equation for analyzing the long-term relationship between variables (See: Table 3). Due to the yearly nature of the series in question, the maximum lag orders are 4 or i = 4. Our model reduced at an order of ARDL by using the Akaike Information Criterion (AIC) to determine the best lag numbers.

**Table 3:** Lag selection criterion.

Lag	LL	LR	df	PP	AIC	HQIC	SBIC
0	−735.844		49	0.000	32.2976	32.4018	32.5758
1	−531.186	409.32	49	0.000	25.5298	26.3638	27.756*
2	−482.986	96.4	49	0.000	25.5646	27.1283	29.7387
3	−391.725	182.52	49	0.000	23.7272	26.0205	29.8492
4	−310.382	162.69*	49	0.000	22.321*	25.344*	30.3908

The estimated F-statistics (See: Table 4) are greater than the higher critical values of I (1) at 1 % significance, which suggests that the null hypothesis that there is no co-integration among the variables should not be accepted. It suggests a long-term relationship between independent variables and economic growth.

**Table 4:** F-bound test for Co-integration relationship.

Null Hypothesis: No levels of relationship				
Test Statistics	Value	significance	I(0)	I(1)
		10 %	2.12	3.23
F-statistics	29.698	5 %	2.45	3.61
		2.5 %	2.75	3.99
K	6	1 %	3.15	4.43

### 4.3 Long run model estimation

As long as co-integration is confirmed, we are permitted to estimate the long-run relationship between the variables. It is also important to estimate the short-run model. Table 5 displays the model's long-run and short-run estimations.

**Table 5:** Long run and Short run model for FDI and Agriculture Sector Relationship.

	(1)		
	D.ln_AFF		
	ADJ	LR	SR
L.ln_AFF	−0.225***		
FDI		−0.526**	
EIG		−0.00671***	
GDP		0.346***	
CPI		0.140***	
TRADE		0.0352**	
GFCF		0.00550	
LD.ln_AFF			−0.311***
L2D.ln_AFF			−0.353***
L3D.ln_AFF			−0.0979
D.GDP			−0.0406***
D.CPI			−0.0210***
LD.CPI			−0.00951*
D.TRADE			−0.0175***
LD.TRADE			−0.0240***
L2D.TRADE			−0.00561
D.GFCF			0.000134
LD.GFCF			−0.000407
L2D.GFCF			−0.0249***
_cons			4.644***
*N*	50		
*R*^2^	0.966		

*p < 0.05, **p < 0.01, ***p < 0.001.

According to the findings of the diagnostic checks, independent factors account for around 96 % of variations in agricultural productivity. Given the significant p-value, the independent variables are generally significant (0.000). Our model is quite reliable, as evidenced by the findings of the diagnostic tests for residual serial correlation and heteroskedasticity. Turning to the parameters, we found that FDI has a negative impact on the agricultural sector and is significant at the 1 % threshold of significance. More specifically, when FDI increases by 1 %, the value added to the agriculture sector decreases by 0.52 %. This negative result is supported by Refs. [9,11,28]. The short-run model is quite compatible with long-run estimation. All the variables in the short run have a significant level of less than 1 %, 5 %, and 10 %. In the short run, there is no relationship between FDI and the Agriculture sector [29]. ECM (−1) determined that the error correction term, which measures how quickly the short-run model moves toward long-run equilibrium, the ECM is negative and statistically significant. In actuality, this is consistent with theory postulates. The conclusion demonstrates that quarterly around 22 % of the short-run volatility would be corrected toward long-run equilibrium.

### 4.4 Diagnostic tests

To check the validity of our estimated model, different diagnostic tests are conducted. Some of the tests which have been performed in our study are represented by table number 6. All the abbreviation results are given elaborately in Table 7 to Table 10 in the appendix section.

All the tests passed their conditions (See: Table 6). That means there is no omitted value, no heteroscedasticity, no autocorrelation, and no multicollinearity problem. Therefore, we can say that the dataset is fit for our model.

**Table 6:** Diagnostic tests.

Name of Test	Value
Ramsey RESET Test	Prob. 0.2370
The BPG test for Heteroscedasticity	Prob. 0.4306
Durbin-Watson Test	1.91886
VIF	3.28

### 4.5 Key findings

This paper has looked at how foreign direct investment has affected the agriculture sector from 1972 through 2021. To examine the long-term and short-term relationship between the researched variables, we used the ARDL Bounds to test this objective. The findings of the study can be summarized with the results of Tables 6 and 7 and also regarding the research Questions of our study. The main findings of the study are that Foreign Direct Investment has no relationship with the agricultural sector in our country in the short run, according to previous literature [24,26,29] and long-run has a negative and significant relationship according to Refs. [9,11,25,28]. Another variable has shown different types of relationships that are not our core findings. This result shows that FDI has no relationship with short-term influence, according to Ref. [26], it supports only the short-run and [29], and negative significant long-term influence on the agricultural sector according to Ref. [9] it supports the long-run part. These findings have occurred because of many reasons. The law of diminishing marginal utility of the agricultural sector, and our country's climate situation, both are the most harmful obstacles. A comprehension of the likely causes of this awful situation could serve as the foundation for the creation of strategic strategies intended to turn the situation around. This undesirable development unquestionably has ramifications for policy.

## 5 Conclusion

We estimate our time series data and detect the negative relationship between FDI and the Agricultural sector in the long run and there is no relationship in the short run. The agricultural sector is an asset for any developing and high-density country because it causes economic growth provides food security and helps to reduce poverty. Bangladesh is a populous country. People need food security for proper agricultural production.

To remove the negative relation in the long run in FDI, the policymakers of Bangladesh should improve control of the corruption system by assuring transparency, taking agriculture-friendly policies, and adopting some training facilities for the farmer to increase their farming skills, and to make sure that FDI inflows into agriculture, and the whole economy. This study is limited to the availability of the data and this research did not receive any funding.

## Data availability statement

The authors do not have permission to share data.

## CRediT authorship contribution statement

**Zakia Sultana:** Writing – original draft, Methodology, Formal analysis, Data curation. **Md Nazmus Sadekin:** Writing – review & editing, Supervision, Software, Resources, Conceptualization.

## Declaration of competing interest

We declare that this manuscript is original, has not been published before, and is not currently being considered for publication elsewhere. We have no conflicts of interest associated with this publication.

## Figures and Tables

**Table 7:** Durbin-Watson Test

Durbin-Watson d-statistic (20, 46) = 1.91886

**Table 8:** The BPG test for Heteroscedasticity

White's test for Ho: homoskedasticity	df	p
against Ha: unrestricted heteroskedasticity		
chi2(45) = 46.00		
Prob > chi2 = 0.4306		
Cameron & Trivedi's decomposition of the IM test		
chi2		
46.000	45	0.431
13.580	19	0.808
1.840	1	0.175
61.420	65	0.603

**Table 9:** Multicollinearity Test

Variance inflation factor		
	VIF	1/VIF
TRADE	6.429	.156
FDI	4.784	.209
GFCF	3.383	.296
CPI	1.919	.521
EIG	1.851	.54
GDP	1.321	.757
Mean VIF	3.281	.

**Table10:** Ramsey RESET Test

Ramsey RESET test using powers of the fitted values of ln_AFF
Ho: The model has no omitted variables
F(3, 40) = 1.47
Prob > F = 0.2370
